# Analysis of the Clinical Efficacy of Azacytidine + Venetoclax in the Treatment of Elderly Patients with Relapsed Refractory Acute Myeloid Leukemia

**DOI:** 10.1155/2022/8691835

**Published:** 2022-10-14

**Authors:** Wei Wang, Quanfang Luo, Qinpin Chen, Aiping Pang, Kuiyan Fang

**Affiliations:** Department of Hematology, Nanxishan Hospital of Guangxi Zhuang Autonomous Region, Guilin, Guangxi Province, China

## Abstract

**Objective:**

To explore the clinical efficacy of azacytidine + venetoclax in the treatment of elderly patients with relapsed refractory acute myeloid leukemia (AML).

**Method:**

The present study included 20 elderly patients with relapsed refractory AML from January 2019 to January 2021. These patients were randomized into treatment groups (*n* = 10, azacytidine alone) and control groups (*n* = 10, azacytidine + venetoclax) by a random number table. The differences in efficacy, adverse reactions, hematology parameters, and immune functions in elderly patients with relapsed refractory AML in two groups were analyzed.

**Results:**

The total efficiency for elderly patients with relapsed refractory AML was 90.00% and significantly higher than that in the control group (40.00%), *P* < 0.05; PLT and WBC after treatment in the treatment group were significantly higher than those in the control group, and Hb was significantly lower than in the control group, *P* < 0.05; CD4+, CD3+, and CD4+/CD8+ after treatment in both groups were significantly lower than those before treatment, *P* < 0.05; CD4+, CD3+, and CD4+/CD8+ after treatment were not significantly different between the two groups, *P* > 0.05; the incidences of adverse reactions were not significantly different between the two groups, *P* > 0.05.

**Conclusion:**

Azacytidine + venetoclax in the treatment of elderly patients with relapsed refractory AML could improve efficacy and hematology parameters with high safety, which is of great significance.

## 1. Introduction

AML is a hematological malignancy. The main feature of AML patients is the clonal proliferation of undifferentiated or abnormally differentiated myeloid cells in the peripheral blood and bone marrow [1, 2]. AML can cause fever, infection, hemorrhage, and anemia, damage the patient's health and even threaten the patient's life. Thus, effective measures are necessary to improve the prognosis [3–5]. Venetoclax is a selective small molecule inhibitor of B-cell lymphoma factor-2 (Bcl-2) and is used in combination with demethylated drugs in the treatment of AML [6, 7]. Azacytidine is a DNA-demethylation drug for AML and is effective in the treatment of relapsed refractory AML [8, 9]. In order to explore the clinical efficacy of azacytidine + venetoclax in the treatment of elderly patients with relapsed refractory AML, the present study included 20 elderly patients with relapsed refractory AML from January 2019 to January 2021 to analyze and clinical value of azacytidine + venetoclax was summarized.

## 2. Information and Methods

### 2.1. Information

The present study included 20 elderly patients with relapsed refractory AML from January 2019 to January 2021.

These patients were randomized into treatment groups (*n* = 10) and control groups (*n* = 10) by a random number table.

Inclusion criteria: a: diagnosed as relapsed refractory AML per criteria for diagnosis and efficacy of hematological diseases; b: and aged ≥60 years old; c: normal liver, kidney, and heart functions; d: good compliance.

Exclusion criteria: a: comorbid with other tumors; b: central nervous system is invaded; c: history of drug allergy.

All patients signed informed consent and this study was approved by the Ethics Committee.

### 2.2. Methods

Patients in the treatment group received azacytidine + venetoclax. Cycle 1, azacytidine, 75 mg/m^2^, sc, days 1–7; venetoclax, day 1, 100 mg, day 2, 200 mg, days 3–28, 400 mg, po. A cycle consists of 28 days. The dosage and administration of azacytidine in subsequent cycles were the same as in cycle 1. The dosage of venetoclax was 400 mg from day 1 to the end of the cycle, po. Patients in the control group received azacytidine alone. The regimen of azacytidine is referred to the treatment group.

Patients in both groups received alkalization and hydration during the treatment to prevent tumor lysis syndrome. Patients with high WBC were orally administered hydroxyurea. Subsequent treatment could be continued only when WBC dropped to <20 × 10^9^/L.

### 2.3. Measurements

The efficacy and adverse reactions in both groups were observed. The differences in hematological parameters and immunological parameters before and after the treatment were analyzed.

Efficacy: complete response (CR): PLT in peripheral blood >100 × 10^9^/L, neutrophils >1.5 × 10^9^/L, proportion of bone marrow blast cells <0.05, no leukemia cells in differential blood count; partial response (PR): neither PLT nor neutrophils in peripheral blood meets the criteria of CR, proportion of bone marrow blast cells is 0.05–0.25 and drops by >50% than that before the treatment; no response (NR): these criteria are not met; the sum of the CR rate and the PR rate is the total efficiency.

Adverse reactions: mainly nausea, vomiting, pulmonary infection, fever, and lower PLT.

Hematology parameters: Venous blood samples of 5 ml were collected from fasting patients. Serum was collected after centrifugation. A hematology analyzer was used to measure PLT count, Hb, and WBC count.

Immunological parameters: CD4+, CD3+, and CD4+/CD8+ measured by flow cytometry.

Data were collected before and after the treatment.

### 2.4. Statistical Analysis

Statistical analysis was performed with SPSS 21.0. Enumeration data were represented by *n* (%) and analyzed by chi-square test. Measurement data were represented by mean ± SD and analyzed by Student's *t*-test. *P* < 0.05 indicated statistical significance.

## 3. Results

### 3.1. General Information

In the treatment group, the mean age was 70.21 ± 8.39 years (60–83 years), including two M0 patients, three M2 patients, three M4 patients, two M5 patients, and five males and five females. In the control group, the mean age was 70.44 ± 7.61 years (61–82 years), including two M0 patients, three M2 patients, two M4 patients, three M5 patients, and 6 males and 4 females. Basic information of elderly patients with relapsed refractory AML in two groups were not significantly different (*P* > 0.05), indicating comparability between the two groups.  Table 1

### 3.2. Efficacy

As shown in Table 2, total efficiency for elderly patients with relapsed refractory AML in the treatment group was 90.00% and significantly higher than that in the control group (40.00%), *P* < 0.05.

### 3.3. Hematology Parameters

As shown in Table 3, PLT and WBC after treatment in both groups were significantly higher than those before treatment, and Hb after treatment was significantly lower than that before the treatment, *P* < 0.05; PLT and WBC after treatment in the treatment group were significantly higher than those in the control group, and Hb was significantly lower than that in the control group. All the differences were significant, *P* < 0.05.

### 3.4. Immunological Parameters

As shown in Table 4, CD4+, CD3+, and CD4+/CD8+ after the treatment in both groups were significantly lower than those before the treatment, *P* < 0.05; CD4+, CD3+ and CD4+/CD8+ after treatment were not significantly different between two groups, *P* > 0.05.

### 3.5. Adverse Reactions

As shown in Table 5, the incidences of adverse reactions between two groups were not significantly different (*P* > 0.05).

## 4. Discussion

The incidence of relapsed refractory AML in the elderly is relatively high. This disease will damage the patient's physical and mental health with a high mortality and poor prognosis [10]. Thus, effective treatment is necessary to improve the prognosis for patients with relapsed refractory AML.

In the present study, total efficiency for elderly patients with relapsed refractory AML was 90.00% and significantly higher than that in the control group (40.00%), *P* < 0.05; PLT and WBC after treatment in the treatment group were significantly higher than those in the control group, and Hb was significantly lower than in the control group, *P* < 0.05; CD4+, CD3+, and CD4+/CD8+ after the treatment in both groups were significantly lower than those before the treatment, *P* < 0.05; CD4+, CD3+, and CD4+/CD8+ after treatment were not significantly different between the two groups, *P* > 0.05; the incidences of adverse reactions were not significantly different between two groups, *P* > 0.05. This indicated that azacytidine + venetoclax for elderly patients with relapsed refractory AML could improve efficacy and hematology parameters, have little effect on immunological parameters, and would not increase the incidence of adverse reactions. Venetoclax is a selective Bcl-2 inhibitor that can bind to Bcl-2 protein, promote the release of proapoptosis Bax and Bim, change the permeability of the mitochondrial outer membrane, activate caspase, and recover the patient's apoptosis [11, 12]. Venetoclax has certain efficacy in the treatment of elderly patients with relapsed refractory AML, yet the efficacy of venetoclax alone is not ideal. Azacytidine is a cytidine analogue. When it binds to RNA and DNA, it has cytotoxicity and specific inhibition on cell cycle; when it binds to DNA methyltransferase, it inhibits methylation of newly synthesized DNA and further promotes recovery of hematopoietic stem cell function [11]. Azacytidine can regulate the differentiation of leukemia cells and induce apoptosis of leukemia cells [12]. Azacytidine is an inhibitor of DNA methyltransferase and can increase the sensitivity of AML to drugs and efficacy [13]. In terms of deficiencies, the current evidence is inadequate to definitively conclude because this study was a single-center study with a relatively small sample size and a relatively short duration of follow-up.

Overall, azacytidine + venetoclax in the treatment of elderly patients with relapsed refractory AML can increase efficacy, improve immunological parameters, and will not increase the incidence of adverse reactions, thus making it worthy of application to improve the prognosis of elderly patients with relapsed refractory AML.

## Figures and Tables

**Table 1:** General information.

Item	Treatment group (*n* = 10)	Control group (*n* = 10)	*χ * ^2^/*t*	*P*
Gender			0.202	0.653
Male	5 (50%)	6 (60%)		
Female	5 (40%)	4 (40%)		
Age (years old)	70.21 ± 8.39	70.44 ± 7.61	0.064	0.949

Classification			0.400	0.940
M0	2 (20%)	2 (20%)		
M2	3 30%)	3 (30%)		
M4	3 (30%)	2 (20%)		
M5	2 (20%)	3 (30%)		

**Table 2:** Efficacy [*n* (%)].

Group	*n*	CR	PR	NR	Total efficiency
Treatment group	10	3 (30.00)	6 (60.00)	1 (10.00)	9 (90.00)
Control group	10	1 (10.00)	3 (30.00)	6 (60.00)	4 (40.00)
*X* ^2^	—	—	—	—	5.495
*P*	—	—	—	—	0.019

**Table 3:** Hematology parameters ($\bar{x}\pm s$).

Group	*n*	PLT (×10^9^/L)		Hb (g/L)		WBC (×10^9^/L)	
		Before	After	Before	After	Before	After
Treatment group	10	71.23 ± 5.69	239.45 ± 32.05	90.45 ± 6.98	74.29 ± 5.14	2.36 ± 0.29	5.71 ± 0.89
Control group	10	70.89 ± 7.02	202.18 ± 20.36	90.22 ± 7.03	79.63 ± 3.20	2.41 ± 0.33	4.40 ± 0.78
*T*	—	0.119	3.104	0.073	2.789	0.360	3.500
*P*	—	0.907	0.006	0.942	0.012	0.723	0.003

**Table 4:** Immunological parameters ($\bar{x}\pm s$).

Group	*n*	CD4+ (%)		CD3+ (%)		CD4+/CD8+	
		Before	After	Before	After	Before	After
Treatment group	10	36.89 ± 2.34	31.56 ± 5.78	50.26 ± 5.45	38.45 ± 5.16	1.50 ± 0.26	1.32 ± 0.25
Control group	10	37.01 ± 1.69	32.02 ± 6.41	49.78 ± 4.32	39.02 ± 4.47	1.52 ± 0.31	1.34 ± 0.29
*T*	—	0.131	0.169	0.218	0.264	0.156	0.165
*P*	—	0.897	0.868	0.830	0.795	0.878	0.871

**Table 5:** Adverse reactions [*n* (%)].

Group	*n*	Nausea and vomiting	Pulmonary infection	Fever	Lower PLT	Total
Treatment group	10	2 (20.00)	1 (10.00)	1 (10.00)	1 (10.00)	5 (50.00)
Control group	10	2 (20.00)	1 (10.00)	2 (20.00)	1 (10.00)	6 (60.00)
*X* ^2^	—	—	—	—	—	0.202
*P*	—	—	—	—	—	0.653

## Data Availability

The analysed data sets generated during the study are available from the corresponding author on reasonable request.
